# Cervical type AB thymoma (Mixed) tumour diagnosis in a mynah as a model to study human: clinicohistological, immunohistochemical and cytohistopathological study

This article has been retracted.

**DOI:** 10.1186/1746-1596-8-98

**Published:** 2013-06-18

**Authors:** Fariba Khaki, Javad Javanbakht, Farhang Sasani, Mohammad Javad Gharagozlou, Alimohammad Bahrami, Hemmat Moslemzadeh, Reza Sheikhzadeh

**Affiliations:** 1 Department of Pathology, Faculty of Veterinary Medicine, Tehran University, Tehran, Iran; 2 Faculty of Para-Veterinary Medicine, University of Ilam, Ilam, Iran; 3 Graduate, Faculty of Veterinary Medicine, Urmia University, Urmia, Iran; 4 Faculty of Veterinary Medicine, Teharn University, Tehran, Iran

**Keywords:** Thymoma, Lymphocytic type, Diagnosis, Mynah,Neck

## Abstract

**Abstract:**

Thymoma is a primary mediastinal neoplasm arising from or exhibiting differentiation towards thymic epithelial cells, typically with the presence of non-neoplastic lymphocytes. A 13-year-old male Mynah bird (*acridotheres tristis*) was presented for evaluation of a 2.3 × 1.5 × 1.0 cm mass in the left ventrolateral cervical region. The clinical signs, radiology, cytohistopathology and immunohistochimy findings related to the thymoma are presented. These findings indicated that the tumor was a type AB thymoma according to the World Health Organization (WHO) and veterinary classification. Thymomas are rarely reported in avian species and this is the first report in a Mynah bird.

**Virtual slides:**

The virtual slide(s) for this article can be found here: http://www.diagnosticpathology.diagnomx.eu/vs/1159525819982779.

## Background

Thymomas are rare malignancies both in human and veterinary medicine. They have been described in a wide range of domestic and laboratory animals, such as rats and mice [1,2], and occur more frequently in older animals. In humans, thymomas usually present in the fourth to fifth decade but can occur at all ages without sex predisposition [3]. In dogs and cats, thymomas are also found in older animals [4], and they are rarely reported in avian species and have only been documented in an African grey parrot (*Psittacus erithacus*),[5] a finch (unspecified species), [6] domestic chickens,[7,8] a budgerigar (*Melopsittacus undulatus*), [9] and a Java sparrow (*Padda oryzivora*) [10].

The etiology of thymomas is not yet understood. In contrast to lymphomas, there is no evidence of a etiology of thymomas in humans and domestic animals. A single report exists that describes a family with high incidence of thymomas and might point to a genetic predisposition [11].

Thymomas are derived from thymic epithelium with variable benign lymphocytic infiltration and thus are classified as lymphocyte-predominant, epithelial-predominant, or mixed [12,13]. Type AB thymoma (also known as mixed thymoma) accounts for approximately 28% to 34% of all thymomas [14,15]. Approximately 16% of this type may be associated with myasthenia gravis [14]. Morphologically, type AB thymoma is a thymic tumor in which foci having the features of type A thymoma are admixed with foci rich in nonneoplastic lymphocytes.[16]. Histologically, these tumors are composed of neoplastic thymic epithelial cells and a variable number of lymphocytes leading to a myriad of histologic subtypes depending on the proportion of these elements [17]. This report describes the clinical signs, cytopathological and immunohistichemical characteristics of a thymoma in a Mynah bird and because there is no established classification of thymic neoplasms in veterinary medicine and the avian thymomas bore a striking resemblance to their human counterparts, an attempt to classify this neoplasm according to the new World Health Organization (WHO) classification of human thymic epithelial tumors was made.

### Case presentation

In April 2013, a 13-year-old adult male red-tail common Mynah bird (*Acridotheres tristis*) was referred to the Avian and Exotics Service of the Tehran Veterinary College, University of Tehran, for evaluation of a firm, round and circular neck mass, off-white to gray, lightly encapsulated, moveable, attached to the underlying tissue and measured 2.3 × 1.5 × 1.0 cm diameter was palpated on the left ventrolateral side of the neck near the thoracic inlet. No evidence of pain or discomfort was noticed, and the bird did not experience any difficulty in prehension and swallowing its food or in breathing. It had been fed predominantly a seed-based and table-food diet. Its owner first noticed the mass 4 weeks before presentation and had progressively increased in size over that period. On gross examination, The bird had lost over 12% of its body weight over the 1 months, decreasing from 184 g to 162 g, because of the size of the mass and the bird's weight loss, and the bird appeared emaciated.

On radiographs, degenerative changes in right tarsal joint and inflammation of its adjacent soft tissues accompanying mineralization of its external soft tissue were observed. In addition, hepatomegaly was recorded as well.

A fine-needle aspirate of the mass was done, and a blood sample was collected for a complete blood cell count (CBC) and plasma biochemical analysis. Radiographs were taken, and the results showed that the mass was of soft-tissue density. Results of the plasma biochemical profile, including bile acids, were within reference ranges (Animal Health Laboratory, University of Tehran). The CBC results revealed a moderate monocytosis at 2.94 × 10^9^ cells/L [2.94 × 10^3^ cells/dL] (reference range for Amazon parrots: 0–0.4 × 10^9^ cells/L [0–0.4 × 10^3^ cells/dL], Animal Health Laboratory, University of Tehran). Aspiration of the mass revealed a cystic structure and results of cytologic examination of the fluid revealed large numbers of lymphocytes with occasional erythrocytes. The bird died during examination.

Cytology this case demonstrated a mixture of round and oval cells. The cytoplasm was scanty and the cell borders were indistinct. Moderate to marked nuclear pleomorphism (Figure 1A and 1B) was noted in this case. These pleomorphic cells displayed anisonucleosis, irregular nuclear membranes, coarse clumping of chromatin, and prominent nucleoli. Mitoses ranged from scant to frequent.

**Figure 1:** **(A) Fine-needle aspiration of thymoma showing predominately round to oval cells with moderate nuclear atypia in type AB thymoma.** Note thick nuclear membranes and more prominent nucleoli. (**B**): High power view of type AB thymoma .Marked pleomorphism characterized these cells. Few lymphocytes are present.

A midline portion of the mass was processed routinely, embedded in paraffin wax, sectioned at 5 μm, and stained with hematoxylin and eosin. For further study, paraffin sections were stained immunohistochemically with CK 14 and CK18 (Abcam Co., Cambridge, USA) for this case.

For immunohistochemistry, sections from each tumor were mounted on adhesive-coated slides (Superfrost Plus, Menzel-Glaser, Braunschwaig, Germany), processed through xylene, and rehydrated in ethanol. Antigen retrieval was by boiling in a microwave oven (700 W) twice for 5 minutes in Tris–EDTA buffer—1.21 g Tris base (A 1379, Applichem, Darmstadt, Germany) and 0.372 g EDTA (8418, Merck, Darmstadt, Germany)—in 1 liter of distilled water, pH 9. Endogenous peroxidase was blocked with 0.6% (v/v) H_2_O_2_ in Tris-buffered saline (TBS; pH 7.6) for 15 minutes at 20°C before the monoclonal antibodies used included those for CK14 and CK18.

### WHO classification of human thymic epithelial tumors

The classification of human thymic epithelial tumors has its origins in a histiogenetic classification originally proposed by Kirchner and Mueller-Hermelink and others [18-20]. The new WHO classification basically recognizes the same histologic entities but uses an alphanumerical system, i.e., combinations of letters and numbers. Thymomas with spindle, oval-shaped epithelial cells are designated type A, and those with small round epithelial components are designated type B. Tumors combining these features are designated type AB. Nonorganotypic thymic carcinomas are classified as type C thymomas. Type B is further subdivided into B1, B2, and B3 on the basis of increasing epithelial areas and the emergence of nuclear atypia [21,22].

Necropsy examination indicated a thin bird with a foul-smelling oral cavity. Dried serous discharge surrounded the incision. A large necrotic ulcer was present in the esophagus with food and caseous material in the subcutaneous space. No gross perforations of the esophagus were present. The intestines appeared necrotic. The resected mass was greatly expansible, but there was no evidence of local invasion or distant metastasis.

Microscopic findings demonstrated that lobules of small polygonal cells with small round or oval vesicular nuclei and indistinct nucleoli accompanied by a variable amount of lymphocytes and the tumoral cells were circular or round and more comprised of lymphoblasts with extensive mitotic features together with and lymphocyte-poor spindle cells (Figure 2A,2B and 2D). The histiocytes with light nuclei and pink cytoplasms among tumoral lymphoid cells were observed (Figure 3D). The tissue was severely hyperemic and remarkable eosinophils existed among cells together with high number of undifferentiated neoplastic cells (Figure 2C).The necrosis was found in some parts with pyknosis and karyorrhexis. In vessels, the tumoral cells were seen. Numerous eosinophils in vessels indicated eosinophilia, (Figure 3C) and plenty of histiocytes contained hemosiderosis in the tumor.

**Figure 2:** **Mixed thymoma; A and B: the tumoral cells were circular or round and more comprised of lymphoblasts with extensive mitotic cells (H&E;20 μm×100), C: Hyperemic and remarkable eosinophils existed among cells (H&E;50 μm×400) D: Note type A and B components.** (H&E;30 μm×200).

**Figure 3:** **Mix ed thymoma; Immunohistochemical staining mixed thymoma with, CK 14(A) and CK 18 (B) are positive for the round cells of the tumor.** Hematoxylin and eosin staining of tissue and cells sections. (**C**): In vessels, the tumoral cells were seen. Numerous eosinophils in vessels indicated eosinophilia (H&E;20 μ×200). (**D**): The histiocytes with light nuclei and pink cytoplasms among tumoral lymphoid cells were observe. (H&E;25 μm×400).

A microscopic examination showed the tumor to contain round shaped cells with a lymphocyte rich component. In the immunohistochemical study, the round cells of the tumor were all positive for CK 14 (Figure 3A) and CK18 (Figure 3B).

On the basis of this case findings, tumour was classified as AB thymomas by analogy with the WHO classification for human neoplasms. Mixture of lymphocyte-associated small polygonal cells and lymphocyte-poor spindle cells areas in tumor correspond closely to AB areas in human tumuors.

These cytohistopathology and immunohistochemical findings indicated that the tumor was a type AB thymoma according to the World Health Organization and veterinary medicine classification.

## Discussion

Thymomas were tumours arising from or exhibiting differentiation toward thymic epithelial cells. It has been reported that different subtypes of thymoma have multifarious genetic characteristics, recent studies indicated that chromosomal 1 gain plays an significant role in molecular genetic mechanism of thymic epithelium tumors [3,12,23]. In a study, Yuqing et al., 2012 suggested that different genes on chromosome 1 might employ different functions in the generation and development of thymic epithelium tumors [12].

Thymic epithelial tumors are rare both in human and veterinary medicine. To our knowledge, this study describes the largest serial of mixed thymoma observed in Mynah bird. In addition to, a description of the morphologic findings, immunohistochemical and cytohistopathological investigations were performed on this tumor with their human counterparts. Because of the high resemblance of the avian thymomas to their human counterparts, the current human WHO classification for thymic epithelial tumors was used.

The avian thymus gland consists of 7 flattened lobes of tissue that are located bilaterally in the subcutis of the neck adjacent to the trachea [24]. Thus, thymomas in birds occur cranial and ventrolateral to the thoracic inlet. In mammals, the thymus gland is located within the mediastinum in the thoracic cavity [25]. The biological behaviors of thymomas are benign and the neoplasia arises from the epithelial portion of the thymus [26].

In all avian species, the differential diagnosis for a cervical swelling is fairly extensive and includes foreign body reaction, trauma, fungal granuloma, abscess, and neoplasia [5]. In this mynah, cervical swelling was observed 4 weeks before presentation and had progressively increased in size over that period. Radiographs performed at that time demonstrated mineral opacities in the lateral cervical region, and degenerative changes in right tarsal joint and inflammation of its adjacent soft tissues accompanying mineralization of its external soft tissue were observed. In addition, hepatomegaly was recorded as well.

In all previously reported avian thymomas, limited presurgical diagnostics were performed before attempted mass resection. Ideally, a complete diagnostic work-up consisting of complete blood count, plasma biochemical analysis, radiographs, and computed tomography would be performed before surgical exploration.Fine-needle aspirate (FNA) with cytologic evaluation or biopsy are useful diagnostic modalities that can be used for an accurate preoperative diagnosis.

FNA biopsy has gained increasing acceptance as a rapid, noninvasive, and effective diagnostic procedure in the investigation of cervical masses [27,28]. Because thymomas are uncommon neoplasms, experience with the cytologic diagnosis of these tumors is limited. To our knowledge, the correlation between cytologic findings of thymomas and various histologic classification has not been well studied previously. Ali and Erozan [26] found that it was possible to correlate the FNA findings with histologic subtypes determined on resection with adequate well preserved material. In the current study, aspirates with a high L:E ratio had a tendency to belong to predominantly mixed.

Tao et al. [28] suggested a classification based on the size, shape, and pleomorphism of the epithelial component, which has been shown to have prognostic value. Riazmontazer et al. [29] also reported a case of invasive thymoma with atypical cytologic features in the aspirate. They described invasive malignant thymomas with cytologic atypia. Our data generally are compatible with these observations. The more atypical the neoplastic cells are, the more likely the tumor will display aggressive behavior.The cytologic features of thymomas include dual lymphoid and epithelial cellular populations and unique neoplastic tissue fragments that reflect histology and allow their accurate identification.

The cytologic diagnosis of thymoma can be extremely challenging. In part, this is because a technically proficient interventional radiologist is needed, epithelial cells may be difficult to recognize in lymphoid rich aspirate smears, and there is inherent sampling error in a tumor that frequently displays heterogeneous histopathology [16,30].

Immunohistochemistry for cytokeratin is helpful in this case, since the presence of rare epithelial cells in serial sections is suggestive of thymoma [31,32]. Cytokeratin profiles have been established in human medicine for the thymus and thymomas, and have been shown to be clinically useful in determining the invasive potential of these neoplasms [16]. Since a cytomorphologic and histologic classification of thymomas seems not to be a useful prognosticator in animals, the use of a pan-specific cocktail of antibodies for cytokeratins is sufficient for the diagnosis of these tumors in veterinary medicine.

Thymoma should be differentiated from other anterior mediastinal neoplasms with epithelial and/or lymphoid differentiation, including Non-Hodgkin (NHL) and Hodgkin lymphomas, thymic carcinomas, and germ cell malignancies. NHL and Hodgkin lymphoma can be separated from thymoma by their dispersed cell population, distinctive cytologic features, and positive staining for CD45, CD20, CD15, and CD30, and negative staining for CK14,CK18, CK20 respectively. Helpful cytologic and immunocytochemical features in making the diagnosis of thymic carcinoma are clear-cut cytological atypia, absence of immature lymphocytes (CD3 + .CD1a+, CD99+), and expression of CD5 and CD70 by neoplastic epithelial cells [12].

Immunohistochemical markers can be used to differentiate the epithelial cells and lymphocytes, aside from the proportion of both cells type [31].In this case, the round cells of the tumor were all positive for CK 14, CK18 and negative for CK10. Based on the WHO and veterinary classification of thymomas [32], this particular case is categorized as mixed type. Overall, the present study confirms previous observations [29,30] that FNA of anterior mediastinal thymic lesions generally yields adequate cellular tissue with distinct cytologic and immunophenotypic features that enables thymoma diagnosis.

In this case, lymphocytes were present individually or in small clump as lobules of small polygonal cells with small round or oval vesicular nuclei and indistinct nucleoli. The proportion of neoplastic cells and nonneoplastic lymphocytes varies widely between tumors and between different lobules of the same tumor [33-35]. Based on this study, thymomas may be categorized in veterinary medicine as lymphocyte predominant, epithelial predominant, or mixed [32].When lymphocytes predominate, the neoplasm must be differentiated from thymic lymphoma.

Thymomas have been described in different sites of the body. The anterior mediastinum or thoracic inlet is their usual site of occurrence, but these neoplasms can also be seen elsewhere, including the cervical region and posterior mediastinum, with variable compression of adjacent structures such as trachea, esophagus, and mediastinal vessels [32,36]. The majority of the thymomas are benign. Local invasion and metastasis are considered by most authors to be uncommon, with metastases being reported in the pulmonary and pericardial pleura, [37] lung, [32,36] mediastinal lymph node, [35] cervical portion of the thymus, [38] kidney, [32] and uterus. Despite, Marx and Mueller-Hermelink considered human type A and AB thymoma as clinically benign tumours [20].

The thymomas examined in our study showed massive local growth with compression, albeit not invasion, of adjacent organs. Furthermore, lymphatic congestion was seen in the cervical lymph nodes and based on their microscopic features of malignancy tumor (such as areas of high cellularity, cellular pleomorphism, high mitotic index, necrotic foci accompanied by pyknosis and karyorrhexis and high number of undifferentiated neoplastic cells), in this case, the tumor was considered to be malignant in nature.

Limitations of the cytological method include an unproven ability to definitively separate thymoma into specific WHO subtypes using cytology alone, and to determine capsular invasion [16]. Altogether, the present report confirms previous observations [26,27] that fine needle aspiration of cervical thymic lesions generally yields adequate cellular tissue with distinct cytologic, histopathologic and immunophenotypic features that enables thymoma diagnosis.

## Conclusion

Based on this report, we recommend that thymomas be included in the differential diagnosis of neck masses in avian. Because it was highly similar to human thymomas, the new WHO classification for human epithelial thymic tumors was used. The tumor was diagnosed as AB type thymomas, and the WHO nomenclature was found to be highly applicable. The incidence of thymoma in avian is unknown; we hope this will become clearer. To our knowledge, this is the first report of cervical thymoma type AB in a mynah, suggesting that this tumour should be included as a differential diagnosis for neck round and spindle cell tumours. Finally, for understanding of these complex neoplasms and the development of the effective differential diagnosis, further investigation will be needed into the clinical features and the basic science.

## Competing interests

The authors declare that they have no conflict of interest.

## Authors’ contributions

FS and MJG participated in the histopathological evaluation, performed the literature review, acquired photomicrographs and drafted the manuscript and gave the final histopathological diagnosis. JJ performed sequencing alignment and manuscript writing. FK carried out the immunohistochemical stains evaluation. HM, AMB and RS edited the manuscript and made required changes. All authors have read and approved the final manuscript.
